# Modified CPT-TODIM method for evaluating the development level of digital inclusive finance under probabilistic hesitant fuzzy environment

**DOI:** 10.1371/journal.pone.0282968

**Published:** 2023-03-29

**Authors:** Yu Deng, Wenxia Zhang

**Affiliations:** 1 Institute of International Education, Henan University of Animal Husbandry and Economy, Zhengzhou, Henan, China; 2 School of Finance and Accounting, Henan University of Animal Husbandry and Economy, Zhengzhou, Henan, China; Prince of Songkla University, THAILAND

## Abstract

Unlike traditional finance, digital inclusive finance is committed to integrating digital technology with the financial industry to bring groups originally excluded from traditional finance back into formal financial services and provide financial services at reasonable prices and matching needs for all social classes. Digital inclusive finance can effectively reduce the financing costs of SMEs, improve the external financing environment of enterprises, and provide more convenient, equal and perfect financial services for enterprises by using technical support such as "big data + artificial intelligence". The development level of digital inclusive finance is a classical multiple attributes group decision making (MAGDM). The Probabilistic hesitant fuzzy sets (PHFSs), which utilize the possible values and its possible membership degrees to depict decision-makers’ behavior in different conditions, has been paid great attention. Though numerous methods have been applied in this environment since PHFSs has been introduced, there are still new fields to be explored. In this paper, we introduce the Cumulative Prospect Theory TODIM (CPT-TODIM) for probabilistic hesitant fuzzy MAGDM(PHF-MAGDM). Meanwhile, the information of entropy is utilized to calculate the weight of attributes, which is used to improve the classical TODIM method. At last, we utilize a numerical case for evaluating the development level of digital inclusive finance to compare the extended CPT-TODIM method with the classical TODIM method.

## 1. Introduction

When we make decisions, the sufficiency and accuracy of data is necessary. However, we always can’t obtain the definite value in most conditions [1–4]. For example, we can’t use a definite value to depict how comfortable the chair is or how is the weather today. In these conditions, the comfort of the chair and the feel about the weather is a fuzzy expression, which often appears in our daily life. Therefore, in order to make decisions with the fuzzy description, Zadeh [5] first introduced the idea of fuzzy sets, and now this theory is applied in many fields such as the cornerstone for the research and decision making and control. Then the extension of fuzzy set for instance, intuitionistic fuzzy was proposed by Atanassov [6]. With the development of this theory, the idea of the hesitant fuzzy set (HFS) was then proposed by Torra, Narukawa and Ieee [7] to extend the fuzzy set which is to denote the uncertainty caused by hesitation solving the common phenomenon in decision making. In the environment of hesitant fuzzy, the membership degree could be indicated by some possible number. The definition brings about the rapid development of hesitant fuzzy set which has a great breakthrough in decision making. Xia and Xu [8] proposed the hesitant fuzzy element(HFE). Xu and Xia [9] raised the score function, deviation function and the comparison rule for HFEs. Xu and Cai [10] provided the aggregating operators under HFEs. Wan, Zhong and Dong [11] produced the GDM based on multiplicative consistency with hesitant fuzzy preference relations. Xu, Wan and Dong [12] created the hesitant fuzzy programming for hybrid MADM with incomplete attribute weight information. Wan, Qin and Dong [13] created hesitant fuzzy mathematical programming for hybrid MAGDM with hesitant fuzzy truth degrees. Wan, Zou, Zhong and Dong [14] created some new information measures for hesitant fuzzy PROMETHEE method. Nevertheless, HFE can be regarded as a particular equivalent form whose occurring probabilities of the possible value is equal. The probabilistic hesitant fuzzy sets (PHFSs) and the corresponding score function, deviation function and its comparison law were proposed by Xu and Zhou [15]. Moreover, the weighted averaging and geometric operators under PHFSs were built by Xu and Zhou [15]. Then the improved PHFS was introduced by Zhang, Xu and He [16] to give more space of hesitation and the integrations of the improved PHES can be calculated by the improved operators.

A large amount of methods to solve the MADM problem are proposed, like VIKOR method [17–20], MABAC method [21–24], TODIM method [25–27], EDAS method [28–32], MOORA method [33–36] and Taxonomy method [37–39]. Among them, the TODIM method is specific in its piecewise function to denote the distance between two elements. Besides TODIM take the negative and positive attributes into consideration by introducing the parameter in the calculation process. Qin, Liang, Li, Chen and Yu [40] solved the MAGDM problems by using the TODIM method and the triangular intuitionistic fuzzy numbers. Krohling, Pacheco and Siviero [41] utilized the TODIM in intuitionistic fuzzy environment. Zhang and Xu [42] expound the novel measured functions-based TODIM approach under hesitant fuzzy environment. Hanine, Boutkhoum, Tikniouine and Agouti [43] compared the fuzzy AHP and fuzzy TODIM methods to solve landfill location selection problems. Passos, Teixeira, Garcia, Cardoso and Gomes [44] used the TODIM-FSE method solve the oil spill response problems. Tseng, Lin, Tan, Chen and Chen [45] used TODIM method to assess green supply chain under uncertainty environment. Li, Shan and Liu [46] used the extended TODIM method for MAGDM which is with the interval intuitionistic fuzzy sets. Wei, Ren and Rodriguez [47] used the hesitant fuzzy linguistic TODIM method based on a score function to solve MAGDM problems. Liu and Teng [48] used the TODIM method based on 2-Dimension uncertain linguistic variable to solve MAGDM problems. Ren, Xu and Gou [49] used Pythagorean fuzzy TODIM approach to solve MAGDM problems. Zhang, Liu and Shi [50] used the extended TODIM based on neutrosophic numbers. Wei [51] used the TODIM method for picture fuzzy MAGDM problems. Zhang, Du and Tian [52] utilized the TODIM under probabilistic hesitant fuzzy circumstance to promise venture capital project. Zhang, Wang and Wang [53] applied the TODIM method to deal with the MAGDM problems under probabilistic interval-valued hesitant fuzzy environment. With the failure to determine the attribute weight, this method was then improved. Tian, Xu and Gu [54] improved the classical TODIM method by using Cumulative Prospect Theory (CPT).

The connotation of traditional finance generally refers to capital financing, including the financial system consisting of financial instruments, financial activities, financial markets, financial institutions, financial supervision, etc [55, 56]. The biggest drawback of the traditional financial model is the problem of achieving the dual performance goals of economic and social benefits for MSMEs. Under the traditional financial environment, the difficulty of financing and the high cost of financing become the key issues that restrict the further development of MSMEs [57–59]. From the traditional economic theory, the less the capital, the higher the marginal return obtained, but the marginal return curve of capital in the traditional economic theory has changed due to risk uncertainty, information asymmetry, adverse selection and moral hazard, and lack of transaction cost. Based on the above real-life dilemmas and basic theories, inclusive finance has been developed [60, 61]. The concept of "inclusive finance" was introduced and promoted by the United Nations in the International Year of Microcredit (2005), and its key targets include small and micro enterprises, people living in remote areas, rural residents, urban low-income people, poor people, people with disabilities, the elderly and other groups. In 2006, the Blue Book on Inclusive Financial Systems drafted by the United Nations pointed out that developing countries should establish a sustainable financial system through policies and systems that can provide people with appropriate products and services [62–64]. Inclusive finance bridges the shortcomings of traditional finance, providing not only accessible, affordable, comprehensive and sustainable financial services for the disadvantaged groups who lack financial options, but also more extensive, convenient and affordable financial services for the general population; it not only expands the breadth of financial services coverage, but also extends the depth of high-quality financial services. Its ultimate goal is to support the economic growth of enterprises and households, eliminate poverty and inequality, and expand the scope of financial services so that all groups can receive appropriate financial services that match their own needs, which is a dynamic and changing guide for action and reflects the value pursuit of financial activities [62–67]. However, the cost of risk identification, credit records and data acquisition for inclusive finance is high, and the general approach adopted by traditional inclusive finance is often difficult to balance the endogenous requirements of accessibility, affordability, comprehensiveness and commercial sustainability, so for inclusive finance to achieve long-term development, it also needs to find a new breakthrough, so the technology based on digital technology, mobile Internet, cloud computing, artificial intelligence, etc. Digital inclusive finance was born [68–70]. Technological progress is an important force to promote financial innovation. In the last fifteen years, along with the rapid development and universal application of digital technology, the digital inclusive finance model has started to gain wider and wider recognition [71, 72]. Digital inclusive finance is to empower traditional inclusive finance through digital technology to help solve the problems encountered in the "last mile" of financial services, so as to significantly reduce the threshold and cost of financial services, improve the efficiency of financial services, and improve the experience of financial services, thus helping traditional inclusive finance break through the bottleneck of development and solve the problems of accessibility, affordability, comprehensiveness, and commercialization [71–73]. In this way, it can help traditional inclusive finance break through the development bottleneck, address the endogenous requirements of accessibility, affordability, comprehensiveness and commercial sustainability, and accelerate the development process of inclusive finance. Its early manifestation was mainly the internetization of traditional business, i.e., the development of offline business to online with the help of Internet platforms. In recent years, with the rapid development and widespread application of financial technology, financial innovation is no longer the simple "Internet + traditional financial business" at the initial stage, but more often the adjustment and reshaping of new product design or service models driven by non-financial institutions through technological progress and technological innovation, such as the U.S. international trade payment tool Pay Pal is a typical representative of digital financial inclusion innovation that relies on technology-driven solutions to practical scenarios.

The development level of digital inclusive finance is a classical MAGDM. The Probabilistic hesitant fuzzy sets (PHFSs), which utilize the possible values and its possible membership degrees to depict decision-makers’ behavior in different conditions, has been paid great attention. In this paper, CPT-TODIM is built for PHF-MAGDM. Meanwhile, the information of entropy is utilized to calculate the weight of attributes, which is used to improve the classical TODIM method. At last, a numerical case is utilized for evaluating the development level of digital inclusive finance to compare the extended CPT-TODIM method with the classical TODIM method. The main research contributions of this study can be summarized: (1) CPT-TODIM method is built under PHFSs; (2) the CPT-TODIM method is developed to tackle the MAGDM with PHFSs; (3) an empirical application for evaluating the development level of digital inclusive finance is offered to proof the developed method; (4) some comparative studies are provided to give effect to the rationality of the built method. In order to do so, the basic research ideas of this article are as follows: Section 2 introduces the PHFSs briefly. In Section 3, this improved CPT-TODIM method is then applied to solve the PHF-MAGDM. Section 4 demonstrates the case study for evaluating the development level of digital inclusive finance. In the end, the Section 5 shows we draw a conclusion based on the research in this paper.

## 2. Preliminary knowledge

In this section, we review numerous means under the PHFSs circumstance as well as CPT-TODIM method.

### 2.1. PHFSs

#### Definition 1 [15]

Let *G* be a fixed set, a PHFSs on *G* is denoted as follows:

$$L=\{<g,\gamma_{g}(b_{g})>|g\in G\}$$ (1)

where the function *γ*_*g*_(*b*_*g*_) is the set of different numbers in [0,1], which denote the possible membership degree of element *g* in *G* to set *L*, and the *b*_*g*_ describes the probabilistic distribution. *k*_(*g*)_*b*_(*g*)_ is named the probabilistic hesitant fuzzy element (PHFE) and showed as *k*(*b*). PHFE can be denoted by $\gamma (b)=\{k_{p}(b_{p})|p=1,2,\ldots ,\#k\}$, where *b*_*p*_ expresses the probability of the possible value *k*_*p*_ and satisfies $\sum_{p=1}^{\#k}b_{p}=1$, where #*k* denotes the number of the possible values.

Definition 2 [15]

Let *γ*_*g*_, *γ*_1_(*b*_1_) and *γ*_2_(*b*_2_) represent three PHFE, then the following algorithms are obtained:

(1) $\gamma_{1}(b_{1})⊕\gamma_{2}(b_{2})=\cup_{k_{p}\in \gamma_{1},k_{q}\in \gamma_{2},b_{p}\in \gamma_{1},b_{q}\in \gamma_{2}}\{(k_{p}+k_{q}-k_{p}k_{q})(b_{p}b_{q})\}$;

(2) $\gamma_{1}(b_{1})⊗\gamma_{2}(b_{2})=\cup_{k_{p}\in \gamma_{1},k_{q}\in \gamma_{2},b_{p}\in \gamma_{1},b_{q}\in \gamma_{2}}\{k_{p}k_{q}(b_{p}b_{q})\}$;

(3) $\lambda \gamma (b)=\cup_{k_{p}\in \gamma ,b_{p}\in b}\{1-{\left(1-k_{p}\right)}^{\lambda })(b_{p})\}$

(4) ${\left(\gamma (b)\right)}^{\lambda }=\cup_{k_{p}\in \gamma ,b_{p}\in b}\{{\left(k_{p}\right)}^{\lambda }(b_{p})\}$

#### Definition 3 [15]

For a PHFE, the score function of *γ*(*b*) is obtained:

$$s(\gamma (b))=\sum_{p=1}^{\#k}k_{p}b_{p}$$ (2)

where #*k* denotes the value of the diverse membership degrees.

Definition **4 [15]**

For a PHFE, the deviation degree of *γ*(*b*) is obtained:

$$d(\gamma (b))=\sum_{i=1}^{\#k}b_{p}{\left[k_{p}-s(\gamma (b))\right]}^{2}$$ (3)

Then we can compare two different PHFEs *γ*_1_(*b*_1_) and *γ*_2_(*b*_2_):

(1) *γ*_1_(*b*_1_)>*γ*_2_(*b*_2_), if *s*(*γ*_1_(*b*_1_))>*s*(*γ*_2_(*b*_2_))

(2) *γ*_1_(*b*_1_)>*γ*_2_(*b*_2_), if *s*(*γ*_1_(*b*_1_)) = *s*(*γ*_2_(*b*_2_)) and *d*(*γ*_1_(*b*_1_))<*d*(*γ*_2_(*b*_2_))

(3) *γ*_1_(*b*_1_) = *γ*_2_(*b*_2_), if *s*(*γ*_1_(*b*_1_)) = *s*(*γ*_2_(*b*_2_)) and *d*(*γ*_1_(*b*_1_)) = *d*(*γ*_2_(*b*_2_))

(4) *γ*_1_(*b*_1_)<*γ*_2_(*b*_2_), if *s*(*γ*_1_(*b*_1_)) = *s*(*γ*_2_(*b*_2_)) and *d*(*γ*_1_(*b*_1_))>*d*(*γ*_2_(*b*_2_))

#### Definition 5 [52]

Let *γ*_1_(*b*_1_) and *γ*_2_(*b*_2_) be two PHFEs. If #*k*_1_>#*k*_2_, then the number of the #*k*_1_−#*k*_2_ should be added to *γ*_1_(*b*_1_) then we obtain the new *γ*_1_(*b*_1_) with the maximal membership degree with the possibility of zero. The Hamming distance measure *d*(*γ*_1_(*b*_1_),*γ*_2_(*b*_2_)) is calculated:

$$d(\gamma_{1}(b_{1}),\gamma_{2}(b_{2}))=\frac{1}{\#k_{1}}\sum_{f=1}^{\#k_{1}}|b_{1}{}^{f}k_{1}{}^{f}-b_{2}{}^{f}k_{2}{}^{f}|,\#k_{1}=\#k_{2}$$ (4)

where #*k*_1_ expresses the number of the membership degree, *k*_*i*_ represent the different membership degrees in *γ*_1_(*b*_1_), *γ*_*q*_ represents the different membership degrees in *γ*_2_(*b*_2_), *k*_*p*_^*f*^ and *k*_*q*_^*f*^ is the *f*th largest value in *k*_*p*_ and *k*_*q*_ respectively, *b*_*p*_^*f*^ and *b*_*q*_^*f*^ represent the possibility of the different membership degrees.

### 2.2 Some HPFE weighted operators

The probabilistic hesitant fuzzy weighted averaging (PHFWA) operator and the probabilistic hesitant fuzzy weighted geometric (PHFWG) operator is introduced [15].

Definition **6 [15]**

Let *γ*_*f*_(*f* = 1,2,⋯,*ε*) be PHFNs, and the PHFWA operator is shown:

$$PHFWA(\gamma_{1},\gamma_{2},\cdots ,\gamma_{\varepsilon })=\overset{\varepsilon }{\underset{f=1}{⊕}}(\nu_{f}\gamma_{f})$$

$$=\underset{k_{1}\in \gamma_{1},k_{2}\in \gamma_{2},\cdots ,k_{f}\in \gamma_{\varepsilon }}{\cup }\{1-\overset{\varepsilon }{\underset{f=1}{\Pi }}{\left(1-k_{f}\right)}^{\nu_{f}}(b_{1}b_{2}\cdots b_{f})\}$$ (5)

where *ν* = (*ν*_1_,*ν*_2_,⋯,*ν*_*ε*_) is the weight of *γ*_*f*_, and $\sum_{f=1}^{\varepsilon }\nu_{f}=1$, *ν*_*f*_∈[0,1], *b*_*f*_ is the probability of *y*_*f*_.

Definition **7 [15]**

Let *γ*_*f*_(*f* = 1,2,⋯,*ε*) be PHFNs, and the PHFWG operator is shown:

$$PHFWG=(\gamma_{1},\gamma_{2},\cdots ,\gamma_{\varepsilon })=\overset{\varepsilon }{\underset{f=1}{⊕}}{\left(\gamma_{f}\right)}^{\nu_{f}}$$

$$=\underset{k_{1}\in \gamma_{1},k_{2}\in \gamma_{2},\cdots ,k_{f}\in \gamma_{\varepsilon }}{\cup }\{\overset{\varepsilon }{\underset{f=1}{\Pi }}{\left(k_{f}\right)}^{\nu_{f}}(b_{1}b_{2}\cdots b_{f})\}$$ (6)

### 2.3 An extended CPT-TODIM method

In this section, we recommend the cumulative prospect theory (CPT) and classical TODIM method [74] which is applied in the Multiple Attribute Decision Making (MADM) and other area, firstly. Nevertheless, the limit of the classical TODIM method has been revealed that this method is not enough to gain the weight of attributes. Then the extended CPT-TODIM method [54] is proposed to improve the limit.

The multiple attribute decision-making matrix is as follows:

$$R={\left[\begin{array}{ccccc} \gamma_{11} & \ldots & \gamma_{1q} & \cdots & \gamma_{1d}\\ \vdots & \ddots & \vdots & \ddots & \vdots \\ \gamma_{p1} & \cdots & \gamma_{pq} & \cdots & \gamma_{pd}\\ \vdots & \ddots & \vdots & \ddots & \vdots \\ \gamma_{c1} & \ldots & \gamma_{cq} & \cdots & \gamma_{cd} \end{array}\right]}_{c\times d};\;p=1,\ldots ,c,q=1\ldots ,d$$

The matrix $\left[\begin{array}{cccc} e_{1}, & e_{2}, & \cdots , & e_{d} \end{array}\right]$ denotes the weighting vector of attributes, which meet the condition that $\sum_{q=1}^{d}e_{q}=1$.

**Step 1.** Figure out the transformed probability of the alternative *O*_*p*_ to *O*_*k*_, according to Eq (7) where *p*,*k*∈*c* and *p*≠*k*

$$\delta_{pkq}(e_{q})=\{\begin{array}{cc} \frac{e_{q}{}^{\eta }}{{\left(e_{q}{}^{\eta }+{\left(1-e_{q}\right)}^{\eta }\right)}^{\frac{1}{\eta }}} & \mathrm{if}\;\gamma_{pq}-\gamma_{kq}\geq 0\\ \frac{e_{q}{}^{\mu }}{\left({\left(e_{q}{}^{\mu }+{\left(1-e_{q}\right)}^{\mu }\right)}^{\frac{1}{\mu }}\right)} & \mathrm{if}\;\gamma_{pq}-\gamma_{kq}<0 \end{array}$$ (7)

**Step 2.** Determine the relative weight δ*_pkq_(*e*_*q*_) of the alternative *O*_*p*_ to *O*_*k*_ by Eq (8)

$$\delta^{*}{}_{pkq}(e_{q})=\frac{\delta_{pkq}(e_{q})}{\max(\delta_{pkq}(e_{l}))}\;q,l\in d$$ (8)

**Step 3.** Count the relative dominance of alternative *O*_*p*_ to *O*_*k*_ underneath the attribute *q* according to Eq (9)

$$\zeta_{q}(O_{p,}O_{k})=\{\begin{array}{cc} \frac{-\theta (\sum_{q=1}^{d}\delta^{*}{}_{pkq}(e_{q})).|\gamma_{pq}-\gamma_{kq}{|}^{\alpha }}{\delta^{*}{}_{pkq}(e_{q})} & \mathrm{if}\;(\gamma_{pq}-\gamma_{kq})<0\\ 0 & \mathrm{if}\;(\gamma_{pq}-\gamma_{kq})=0\\ \frac{\delta^{*}{}_{pkq}(e_{q}).|\gamma_{pq}-\gamma_{kq}{|}^{\beta }}{\sum_{q=1}^{d}\delta^{*}{}_{pkq}(e_{q})} & \mathrm{if}\;(\gamma_{pq}-\gamma_{kq})>0 \end{array}$$ (9)

where *α*, *β*, *θ* are the arguments.

**Step 4.** Figure out the dominance degree of the alternative *O*_*p*_, over the others by Eq (10)

$$\tau (O_{p})=\sum_{p=1}^{c}{\sum_{q=1}^{d}\zeta }_{q}(O_{p,}O_{k})p=1,2,\ldots ,c$$ (10)

**Step 5**. Calculate the overall dominance degree of the alternative *O*_*p*_, by Eq (11)

$$\psi (O_{p})=\frac{\tau (O_{p})-\underset{p}{\min}(\tau (O_{p}))}{\underset{p}{\max}(\tau (O_{p}))-\underset{p}{\min}(\tau (O_{p}))}\;p=1,2,\ldots ,c$$ (11)

**Step 6.** Obtain the final ranking of overall dominance degree *ψ*(*O*_*p*_). The greater the value of the overall dominance degree *ψ*(*O*_*p*_) is, the more appropriate the alternative is.

## 3. Extended CPT-TODIM for PHF-MAGDM

The MAGDM matrix $R^{f}={\left[\gamma^{f}{}_{pq}(b_{pq})\right]}_{c\times d}$ is as follows where the alternatives are expressed as *O* = {*O*_1_,*O*_2…,_*O*_*c*_} and the attributes is expressed as *U* = {*U*_1_,*U*_2…,_*U*_*d*_}, and the weight of the attribute is unclear. The set of the decision maker is *D* = {*D*_1_,*D*_2_,…,*D*_*ε*_}, whose weight vector is *ν* = (*ν*_1_,*ν*_2_,⋯,*ν*_*ε*_),(*f* = 1,2,…,*ε*), $\sum_{f=1}^{\varepsilon }\nu_{f}=1$.

Then, the CPT-TODIM is proposed for PHF-MAGDM. The framework is shown in Fig 1.

**Fig 1:** The framework of the probability hesitant fuzzy MAGDM using extended TODIM.

**Step 1.** Normalize the decision matrices.

When *U*_*q*_ is the positive attribute, the normalized probabilistic hesitant fuzzy element is determined by Eq (12)

$$\gamma_{pq}^{*}=\{k_{pq}(b_{pq})\};\;q=1\ldots ,d$$ (12)

When *U*_*q*_ is the negative attribute, the normalized probabilistic hesitant fuzzy element is determined by Eq (13)

$$\gamma_{pq}^{*}=\{(1-k_{pq})(b_{pq})\};\;q=1,\ldots ,d$$ (13)

*γ*_pq_* represents the value of normalized decision matrix.

For two PHFEs, the value of #*k*_1_ and #*k*_2_ may be different from each other. Assume #*k*_1_>#*k*_2_, then we can add the number of #*k*_1_−#*k*_2_ different membership degree to *k*_2_(*b*_2_). We add the maximal membership degree to *k*_2_(*b*_2_), with the value of possibility of it is 0. Then the decision matrix can be normalized like that.

**Step 2.** Aggregate the information to synthesize PHFE decision matrices by using the PHFWA which calculated by Eq (14)

$$PHFWA(\gamma_{1}^{*},\gamma_{2}^{*},\cdots ,\gamma_{\varepsilon }^{*})=\overset{\varepsilon }{\underset{f=1}{⊕}}(\nu_{f}\gamma_{f}^{*})$$

$$=\underset{k_{1}^{*}\in \gamma_{{}_{1}}^{*},k_{2}^{*}\in \gamma_{2}^{*},\cdots ,k_{f}^{*}\in \gamma_{f}^{*}}{\cup }\{1-\overset{\varepsilon }{\underset{f=1}{\Pi }}{\left(1-k_{f}^{*}\right)}^{\nu_{f}}(b_{1}b_{2}\cdots b_{f})\}$$ (14)

**Step 3.** Figure out the distance between $\gamma_{pq}^{*}$ and negative ideal point *γ*^−^

$$d(\gamma_{pq}^{*},\gamma^{-})=\frac{1}{\#k_{1}}\sum_{l=1}^{\#k_{1}}|b_{pq}^{*}k_{pq}^{*}-b^{-}k_{q}^{-}|$$ (15)

**Step 4**. Obtain attributes weights using the Entropy weighting method through Eq (16)

$$e_{q}=\frac{1-g_{q}}{\sum_{q=1}^{d}\left(1-g_{q}\right)}\;q=1,2,\cdots ,d$$ (16)

where *g*_*q*_ represents the entropy of the *q*th attributes and calculate it by Eq (17)

$$g_{q}=-\frac{1}{\ln c}\sum_{p=1}^{c}\left[\frac{d(\gamma_{pq},\gamma_{q}^{-})}{\sum_{p=1}^{c}d(\gamma_{pq},\gamma_{q}^{-})}\ln(\frac{d(\gamma_{pq},\gamma_{q}^{-})}{\sum_{p=1}^{c}d(\gamma_{pq},\gamma_{q}^{-})})\right]$$ (17)

where $\gamma_{q}^{-}$ means the *q*th negative ideal point, $d(\gamma_{pq},\gamma_{q}^{-})$ denotes the distance between *γ*_*pq*_ and $\gamma_{q}^{-}$

**Step 5.** Calculate the transformed probability of the alternative *O*_*p*_ to *O*_*q*_. The equation is Eq (18)

$$\delta_{pkq}(e_{q})=\{\begin{array}{cc} \frac{e_{q}{}^{\eta }}{{\left(e_{q}{}^{\eta }+{\left(1-e_{q}\right)}^{\eta }\right)}^{\frac{1}{\eta }}} & \mathrm{if}\;\gamma_{pq}\geq \gamma_{kq}\\ \frac{e_{q}{}^{\mu }}{\left({\left(e_{q}{}^{\mu }+{\left(1-e_{q}\right)}^{\mu }\right)}^{\frac{1}{\mu }}\right)} & \mathrm{if}\;\gamma_{pq}<\gamma_{kq} \end{array}$$ (18)

where *η*, *μ* are the arguments to describe the curvature of the weighting function

**Step 6.** Obtain the relative weight δ*_pkq_(*e*_*q*_) of the alternative *O*_*p*_ to *O*_*k*_ by Eq (19)

$$\delta^{*}{}_{pkq}(e_{q})=\frac{\delta_{pkq}(e_{q})}{\max(\delta_{pkq}(e_{l}))}\;q,l=1,2,\cdots ,d$$ (19)

**Step 7**. Count the relative dominance of alternative *O*_*p*_ to *O*_*k*_ underneath attribute *q* by Eq (20)

$$\zeta_{q}(O_{p,}O_{k})=\{\begin{array}{cc} \frac{-\theta (\sum_{q=1}^{d}\delta^{*}{}_{pkq}(e_{q})).d{\left(\gamma_{pq},\gamma_{kq}\right)}^{\alpha }}{\delta^{*}{}_{pkq}(e_{q})} & \mathrm{if}\;\gamma_{pq}-\gamma_{kq}<0\\ 0 & \mathrm{if}\;\gamma_{pq}-\gamma_{kq}=0\\ \frac{\delta^{*}{}_{pkq}(e_{q}).d{\left(\gamma_{pq},\gamma_{kq}\right)}^{\beta }}{\sum_{q=1}^{d}\delta^{*}{}_{pkq}(e_{q})} & \mathrm{if}\;\gamma_{pq}-\gamma_{kq}>0 \end{array}$$ (20)

where *α*, *β*, *θ* are the arguments.

**Step 8**. Figure out the dominance degree of alternative *O*_*p*_ over the other alternatives by Eq (21)

$$\tau (O_{p})=\sum_{k=1}^{c}\sum_{q=1}^{d}\zeta_{q}(O_{p,}O_{k})\;p=1,2,\ldots ,c$$ (21)

**Step 9.** Calculate the overall dominance degree of the alternative *O*_*p*,_ by Eq (22)

$$\psi (O_{p})=\frac{\tau (O_{p})-\underset{p}{\min}(\tau (O_{p}))}{\underset{p}{\max}(\tau (O_{p}))-\underset{p}{\min}(\tau (O_{p}))}\;p=1,2,\ldots ,c$$ (22)

**Step 10.** Obtain the final rank of overall dominance degree *ψ*(*O*_*p*_). The greater the value of the overall dominance degree *ψ*(*O*_*p*_) is, the more appropriate the alternative is.

## 4. Numerical examples

### 4.1 Numerical example

The report of the 19th Party Congress clearly points out that "deepening the reform of the financial system and enhancing the capacity of financial services for the real economy", and requires that "efforts should be made to accelerate the construction of an industrial system with synergistic development of the real economy, science and technology innovation, modern finance and human resources". The government’s work report for 2021 also calls for "accelerating digital development, creating new advantages in the digital economy, collaborating to promote digital industrialization and digital transformation of industries, accelerating the pace of building a digital society, improving the level of digital government construction, creating a good digital ecology, and building a digital China", while clearly proposing that "large At the same time, it is clearly proposed that "the loans of large commercial banks for small and medium-sized enterprises will increase by more than 30%" [55, 56, 75, 76]. "The 14th Five-Year Plan emphasizes "accelerating digital development, building a digital China, and promoting the deep integration of digital technology and the real economy", and points out that "a modern financial system with a high degree of adaptability, competitiveness and inclusiveness will be improved. It also points out that "to improve a modern financial system that is highly adaptable, competitive and inclusive, and to build an institutional mechanism for effective financial support for the real economy", and clearly calls for "enhancing financial inclusion". In recent years, digital inclusive finance has received wide attention from all walks of life. On the one hand, traditional financial institutions represented by commercial banks, securities companies and insurance companies have encountered unprecedented challenges under the impact of Internet finance and difficulties and obstacles in the development of inclusive finance, which urgently need to be solved by modern information technology such as big data, blockchain, cloud computing and mobile communication technology; on the other hand, non-banking financial institutions such as microfinance companies and consumer finance companies have been taking inclusive finance as a priority [77–79]. On the other hand, non-bank financial institutions such as microfinance companies and consumer finance companies have been taking inclusive finance as one of the important areas for business expansion and innovation, but due to the limitations in capital scale, risk management and financial regulation, such non-bank financial institutions cannot fully meet the financing needs of SMEs [62, 80, 81]. The Internet and digital technology provide a new path for business model change, through which the capacity of inclusive financial services can be enhanced. the digital inclusive finance index grew at an average annual rate of 29.1% during the ten-year period from 2011 to 2020, but due to the development so far, the coverage of the population has been extensive, and the growth rate of the digital inclusive finance index has slowed down in the past three years [63, 64, 82]. The development level evaluation of digital inclusive finance is a classical MAGDM. In this paper, the CPT-TODIM is built for PHF-MAGDM. Then, a numerical case is given for evaluating the development level of digital inclusive finance. And there are five digital inclusive finance cities *O*_*p*_(*p* = 1,2,3,4,5) to be chosen. The management departments adopt six attributes to assess the development level of these five digital inclusive finance cities:(1) *U*_1_ is the financial service cost,(2) *U*_2_ is the financial service accessibility,(3) *U*_3_ is the digital financial price,(4) *U*_4_ is the depth of digital financial usage, (5) *U*_5_ is the financial service quality (6) *U*_6_ is the breadth of digital financial coverage. Except for (1) and (3) is the negative attributes, the others are positive attributes. The three experts’ weights are *ν* = (*ν*_1_,*ν*_2_,*ν*_3_)^*T*^ = (0.38,0.41,0.21)^*T*^. Then the PHF decision matrices which are given by the three experts are shown in Tables 1–3.

**Table 1:** PHF matrix *R*_1_ given by the first expert.

	*U*_1_	*U*_2_	*U*_3_	*U*_4_	*U*_5_	*U*_6_
*O*_1_	{0.3(0.2), 0.4(0.8)}	{0.2(0.3), 0.7(0.7)}	{0.1(0.5), 0.2(0.5)}	{0.4(0.2), 0.6(0.8)}	{0.2(1)}	{0.2(0.3), 0.7(0.7)}
*O*_2_	{0.4(0.2), 0.6(0.8)}	{0.3(0.5), 0.6(0.5),}	{0.2(0.2), 0.4(0.8)}	{0.6(0.6), 0.4(0.4),}	{0.2(0.4), 0.5(0.6)}	{0.4(0.2), 0.1(0.8)}
*O*_3_	{0.2(1)}	{0.2(0.1), 0.4(0.9)}	{0.3(0.4), 0.4(0.6)}	{0.4(0.2), 0.8(0.8)}	{0.3(0.6), 0.5(0.4)}	{0.4(0.3), 0.6(0.7)}
*O*_4_	{0.6(0.6), 0.8(0.4)}	{0.6(0.2), 0.8(0.8)}	{0.5(0.4), 0.6(0.6)}	{0.4(0.5), 0.7(0.5)}	{0.1(0.5), 0.3(0.5)}	{0.1(0.1), 0.4(0.9)}
*O*_5_	{0.5(0.1), 0.7(0.9)}	{0.4(0.3), 0.5(0.7)}	{0.5(0.2), 0.7(0.8)}	{0.3(0.1), 0.4(0.9)}	{0.6(0.3), 0.8(0.7)}	{0.5(0.2), 0.7(0.8)}

**Table 2:** PHF matrix *R*_2_ given by the second expert.

	*U*_1_	*U*_2_	*U*_3_	*U*_4_	*U*_5_	*U*_6_
*O*_1_	{0.1(0.3), 0.3(0.7)}	{0.2(0.2), 0.4(0.8)}	{0.4(0.3), 0.6(0.7)}	{0.3(0.2), 0.7(0.8)}	{0.3(0.3), 0.4(0.7)}	{0.2(0.4), 0.7(0.6)}
*O*_2_	{0.3(0.5), 0.6(0.5)}	{0.3}	{0.2(0.2), 0.4(0.8)}	{0.5(0.2), 0.4(0.8)}	{0.2(0.3), 0.5(0.7)}	{0.4(0.2), 0.7(0.8)}
*O*_3_	{0.4(0.2), 0.5(0.8)}	{0.2(0.3), 0.5(0.7)}	{0.2(0.4), 0.5(0.6)}	{0.1(0.2), 0.5(0.8)}	{0.1(0.6), 0.3(0.4)}	{0.5(0.3), 0.7(0.7)}
*O*_4_	{0.3(0.3), 0.6(0.7)}	{0.2(0.2), 0.7(0.8)}	{0.3(0.2), 0.5(0.8)}	{0.2(0.4), 0.8(0.6)}	{0.3(0.5), 0.6(0.5)}	{0.1(0.2), 0.4(0.8)}
*O*_5_	{0.4(0.3), 0.5(0.7)}	{0.2(0.4), 0.6(0.6)}	{0.2(0.1), 0.5(0.9)}	{0.2(0.1), 0.4(0.9)}	{0.5(0.4), 0.6(0.6)}	{0.4(0.3), 0.5(0.7)}

**Table 3:** PHF matrix *R*_3_ given by the third expert.

	*U*_1_	*U*_2_	*U*_3_	*U*_4_	*U*_5_	*U*_6_
*O*_1_	{0.4(0.1), 0.5(0.9)}	{0.2(0.5), 0.7(0.5)}	{0.2}	{0.4(0.4), 0.6(0.6)}	{0.2(0.7), 0.3(0.3)}	{0.2(0.1), 0.4(0.9)}
*O*_2_	{0.2(0.1), 0.4(0.9)}	{0.3(0.7), 0.6(0.3)}	{0.2(0.7), 0.7(0.3)}	{0.3(0.2), 0.7(0.8)}	{0.5(0.9), 0.9(0.1)}	{0.4(0.2), 0.1(0.8)}
*O*_3_	{0.2(0.2), 0.7(0.8)}	{0.4(0.2), 0.8(0.8)}	{0.3(0.4), 0.4(0.6)}	{0.3(0.4), 0.8(0.6)}	{0.3(0.4), 0.5(0.6)}	{0.2(0.1), 0.6(0.9)}
*O*_4_	{0.6(0.2), 0.8(0.8)}	{0.7(0.5), 0.8(0.5)}	{0.3(0.4), 0.6(0.6)}	{0.1(0.2), 0.7(0.8)}	{0.1(0.3), 0.3(0.7)}	{0.1(0.2), 0.4(0.8)}
*O*_5_	{0.4(0.1), 0.8(0.9)}	{0.4(0.3), 0.5(0.7)}	{0.5(0.4), 0.7(0.6)}	{0.3(0.6), 0.4(0.4)}	{0.6(0.4), 0.7(0.6)}	{0.2(0.3), 0.7(0.7)}

Then, the CPT-TODIM method is built to solve the PHF-MAGDM for development level evaluation of digital inclusive finance.

**Step 1.** Use Eq (12) and Eq (13) to transform the negative attributes into positive attributes. The result is shown in Tables 4, 5 and 6.

**Table 4:** Normalize PHF matrix *Y*_1_ given by the first expert.

	*U*_1_	*U*_2_	*U*_3_	*U*_4_	*U*_5_	*U*_6_
*O*_1_	{0.7(0.2), 0.6(0.8)}	{0.2(0.3), 0.7(0.7)}	{0.9(0.5), 0.8(0.5)}	{0.4(0.2), 0.6(0.8)}	{0.2(1), 0.2(0)}	{0.2(0.3), 0.7(0.7)}
*O*_2_	{0.6(0.2), 0.4(0.8)}	{0.3(0.5), 0.6(0.5),}	{0.8(0.2), 0.6(0.8)}	{0.6(0.6), 0.4(0.4),}	{0.2(0.4), 0.5(0.6)}	{0.4(0.2), 0.1(0.8)}
*O*_3_	{0.8(1), 0.8(0)}	{0.2(0.1), 0.4(0.9)}	{0.7(0.4), 0.6(0.6)}	{0.4(0.2), 0.8(0.8)}	{0.3(0.6), 0.5(0.4)}	{0.4(0.3), 0.6(0.7)}
*O*_4_	{0.4(0.6), 0.2(0.4)}	{0.6(0.2), 0.8(0.8)}	{0.5(0.4), 0.4(0.6)}	{0.4(0.5), 0.7(0.5)}	{0.1(0.5), 0.3(0.5)}	{0.1(0.1), 0.4(0.9)}
*O*_5_	{0.5(0.1), 0.3(0.9)}	{0.4(0.3), 0.5(0.7)}	{0.5(0.2), 0.3(0.8)}	{0.3(0.1), 0.4(0.9)}	{0.6(0.3), 0.8(0.7)}	{0.5(0.2), 0.7(0.8)}

**Table 5:** Normalize PHF matrix *Y*_2_ given by the second expert.

	*U*_1_	*U*_2_	*U*_3_	*U*_4_	*U*_5_	*U*_6_
*O*_1_	{0.9(0.3), 0.7(0.7)}	{0.2(0.2), 0.4(0.8)}	{0.6(0.3), 0.4(0.7)}	{0.3(0.2), 0.7(0.8)}	{0.3(0.3), 0.4(0.7)}	{0.2(0.4), 0.7(0.6)}
*O*_2_	{0.7(0.5), 0.4(0.5)}	{0.3(1), 0.3(0)}	{0.8(0.2), 0.6(0.8)}	{0.5(0.2), 0.4(0.8)}	{0.2(0.3), 0.5(0.7)}	{0.4(0.2), 0.7(0.8)}
*O*_3_	{0.6(0.2), 0.5(0.8)}	{0.2(0.3), 0.5(0.7)}	{0.8(0.4), 0.5(0.6)}	{0.1(0.2), 0.5(0.8)}	{0.1(0.6), 0.3(0.4)}	{0.5(0.3), 0.7(0.7)}
*O*_4_	{0.7(0.3), 0.4(0.7)}	{0.2(0.2), 0.7(0.8)}	{0.7(0.2), 0.5(0.8)}	{0.2(0.4), 0.8(0.6)}	{0.3(0.5), 0.6(0.5)}	{0.1(0.2), 0.4(0.8)}
*O*_5_	{0.6(0.3), 0.5(0.7)}	{0.2(0.4), 0.6(0.6)}	{0.8(0.1), 0.5(0.9)}	{0.2(0.1), 0.4(0.9)}	{0.5(0.4), 0.6(0.6)}	{0.4(0.3), 0.5(0.7)}

**Table 6:** Normalize PHF matrix *Y*_3_ given by the third expert.

	*U*_1_	*U*_2_	*U*_3_	*U*_4_	*U*_5_	*U*_6_
*O*_1_	{0.6(0.1), 0.5(0.9)}	{0.2(0.5), 0.7(0.5)}	{0.8(1), 0.8(0)}	{0.4(0.4), 0.6(0.6)}	{0.2(0.7), 0.3(0.3)}	{0.2(0.1), 0.4(0.9)}
*O*_2_	{0.8(0.1), 0.6(0.9)}	{0.3(0.7), 0.6(0.3)}	{0.8(0.7), 0.3(0.3)}	{0.3(0.2), 0.7(0.8)}	{0.5(0.9), 0.9(0.1)}	{0.4(0.2), 0.1(0.8)}
*O*_3_	{0.8(0.2), 0.3(0.8)}	{0.4(0.2), 0.8(0.8)}	{0.7(0.4), 0.6(0.6)}	{0.3(0.4), 0.8(0.6)}	{0.3(0.4), 0.5(0.6)}	{0.2(0.1), 0.6(0.9)}
*O*_4_	{0.4(0.2), 0.2(0.8)}	{0.7(0.5), 0.8(0.5)}	{0.7(0.4), 0.4(0.6)}	{0.1(0.2), 0.7(0.8)}	{0.1(0.3), 0.3(0.7)}	{0.1(0.2), 0.4(0.8)}
*O*_5_	{0.6(0.1), 0.2(0.9)}	{0.4(0.3), 0.5(0.7)}	{0.5(0.4), 0.3(0.6)}	{0.3(0.6), 0.4(0.4)}	{0.6(0.4), 0.7(0.6)}	{0.2(0.3), 0.7(0.7)}

**Step 2.** Calculate the overall decision matrix using Eq (14), and it is shown in Table 7.

**Table 7:** The overall PHF matrix.

	*U*_1_	*U*_2_	*U*_3_	*U*_4_	*U*_5_	*U*_6_
*O*_1_	{0.203(0.006),0.213(0.054),0.319(0.014),0.334(0.126),0.227(0.024),0.237(0.216),0.355(0.056),0.373(0.504)}	{0.800(0.030),0.651(0.030),0.711(0.120),0.579(0.120),0.551(0.070),0.449(0.070),0.490(0.280),0.399(0.28)}	{0.204(0.150),0.241(0.350),0.266(0.150),0.314(0.35)}	{0.639(0.024),0.587(0.036),0.452(0.056),0.415(0.084),0.548(0.096),0.503(0.144),0.387(0.224),0.355(0.336)}	{0.757(0.210),0.736(0.090),0.711(0.490),0.691(0.210)}	{0.800(0.012),0.753(0.108),0.535(0.018),0.504(0.162),0.551(0.028),0.519(0.028),0.519(0.252),0.369(0.042),0.347(0.378)}
*O*_2_	{0.307(0.010),0.355(0.090),0.408(0.010), 0.472(0.090),0.359(0.040),0.415(0.360),0.476(0.040),0.551(0.36)}	{0.700(0.350),0.622(0.150),0.566(0.350),0.503(0.15)}	{0.200(0.028),0.260(0.124),0.266(0.112),0.346(0.496),0.339(0.048),0.45(0.192)}	{0.493(0.024),0.413(0.090),0.531(0.096),0.445(0.384),0.575(0.016),0.481(0.064),0.620(0.064),0.519(0.256)}	{0.725(0.108),0.517(0.012),0.598(0.252),0.426(0.028),0.606(0.162),0.432(0.018),0.500(0.378),0.357(0.042)}	{0.600(0.008),0.653(0.032),0.452(0.032),0.492(0.128),0.700(0.032),0.762(0.128),0.527(0.128),0.574(0.512)}
*O*_3_	{0.266(0.200),0.346(0.160),0.291(0.160),0.379(0.640)}	{0.753(0.006),0.598(0.024),0.621(0.014),0.493(0.056),0.675(0.054),0.536(0.216),0.557(0.126),0.442(0.504)}	{0.254(0.064),0.270(0.096),0.370(0.096),0.393(0.144),0.283(0.096),0.301(0.144),0.413(0.144),0.438(0.216)}	{0.732(0.016),0.563(0.024),0.575(0.064),0.442(0.096),0.482(0.064),0.371(0.096),0.379(0.256),0.291(0.384)}	{0.776(0.144),0.723(0.216), 0.700(0.096),0.652(0.144),0.683(0.096),0.636(0.144),0.616(0.064),0.574(0.096)}	{0.591(0.009),0.511(0.081),0.480(0.021),0.415(0.189),0.507(0.021),0.438(0.189),0.411(0.049),0.355(0.441)}
*O*_4_	{0.452(0.036),0.480(0.144), 0.60(0.0840),0.637(0.336),0.504(0.024),0.535(0.096),0.669(0.056),0.711(0.224)}	{0.500(0.020),0.459(0.020),0.335(0.080),0.307(0.080),0.384(0.080),0.353(0.080),0.257(0.32),0.236(0.32)}	{0.364(0.032),0.421(0.048),0.449(0.128),0.520(0.1920),0.390(0.048),0.452(0.072),0.481(0.192),0.557(0.288)}	{0.735(0.04),0.584(0.160),0.416(0.060),0.331(0.240),0.565(0.040),0.449(0.160),0.302(0.060),0.254(0.240)}	{0.812(0.075),0.770(0.175),0.645(0.075),0.612(0.175),0.738(0.075),0.700(0.175),0.587(0.075),0.556(0.175)}	{0.900(0.004),0.827(0.016),0.762(0.016),0.700(0.064),0.771(0.036),0.709(0.144),0.653(0.144),0.600(0.576)}
*O*_5_	{0.453(0.003),0.504(0.027),0.477(0.007),0.552(0.063),0.495(0.027),0.572(0.243),0.542(0.063),0.627(0.567)}	{0.675(0.036),0.65(0.084),0.508(0.054),0.489(0.126),0.63(0.084),0.606(0.196),0.474(0.126),0.456(0.294)}	{0.343(0.008),0.369(0.012),0.500(0.072),0.537(0.108),0.390(0.032),0.419(0.048),0.568(0.288),0.61(0.432)}	{0.739(0.006),0.716(0.004),0.657(0.054),0.636(0.036),0.697(0.054),0.675(0.036),0.620(0.4860),0.60(0.324)}	{0.438(0.048),0.413(0.072),0.400(0.072),0.377(0.108),0.337(0.112),0.317(0.168),0.307(0.168),0.289(0.252)}	{0.595(0.018),0.484(0.042),0.552(0.042),0.449(0.098),0.490(0.072),0.399(0.168),0.454(0.168),0.370(0.392)}

**Step 3**. Calculate the distance by using Eq (15), and the result is shown in Table 8.

**Table 8:** The distance between $\gamma_{pq}^{*}$ and *γ*^−^.

	*U*_1_	*U*_2_	*U*_3_	*U*_4_	*U*_5_	*U*_6_
$d_{1i^{-}}$	0.000	0.029	0.000	0.010	0.103	0.016
$d_{2i^{-}}$	0.017	0.058	0.042	0.014	0.069	0.031
$d_{3i^{-}}$	0.012	0.031	0.053	0.000	0.050	0.000
$d_{4i^{-}}$	0.036	0.000	0.059	0.015	0.037	0.046
$d_{5i^{-}}$	0.036	0.031	0.072	0.041	0.000	0.023

**Step 4.** Calculate the weights through Eqs (16 and 17):

$$e_{q}=(0.171,0.16,0.154,0.185,0.165,0.165).$$

**Step 5.** Obtain the transformed probability of *O*_*p*_ to the others through Eq (17), (*η* = 0.61, *μ* = 0.69 [83]), the result is shown in Tables 9–13.

**Table 9:** The transformed probability of alternative *O*_1_ to others.

	*U*_1_	*U*_2_	*U*_3_	*U*_4_	*U*_5_	*U*_6_
*δ*_12_	0.234	0.225	0.220	0.246	0.238	0.229
*δ*_13_	0.234	0.234	0.220	0.251	0.238	0.237
*δ*_14_	0.234	0.234	0.220	0.251	0.238	0.237
*δ*_15_	0.234	0.225	0.220	0.246	0.238	0.237

**Table 10:** The transformed probability of alternative *O*_2_ to others.

	*U*_1_	*U*_2_	*U*_3_	*U*_4_	*U*_5_	*U*_6_
*δ*_21_	0.241	0.234	0.230	0.251	0.229	0.237
*δ*_23_	0.241	0.234	0.220	0.251	0.229	0.237
*δ*_24_	0.234	0.234	0.220	0.251	0.229	0.237
*δ*_25_	0.234	0.234	0.220	0.246	0.238	0.237

**Table 11:** The transformed probability of alternative *O*_3_ to others.

	*U*_1_	*U*_2_	*U*_3_	*U*_4_	*U*_5_	*U*_6_
*δ*_31_	0.241	0.225	0.230	0.246	0.229	0.229
*δ*_32_	0.234	0.225	0.230	0.246	0.238	0.229
*δ*_34_	0.234	0.234	0.220	0.246	0.238	0.229
*δ*_35_	0.234	0.225	0.220	0.246	0.238	0.229

**Table 12:** The transformed probability of alternative *O*_4_ to others.

	*U*_1_	*U*_2_	*U*_3_	*U*_4_	*U*_5_	*U*_6_
*δ*_41_	0.241	0.225	0.230	0.246	0.229	0.229
*δ*_42_	0.241	0.225	0.230	0.246	0.238	0.229
*δ*_43_	0.241	0.225	0.230	0.251	0.229	0.237
*δ*_45_	0.241	0.225	0.220	0.246	0.238	0.237

**Table 13:** The transformed probability of alternative *O*_5_ to others.

	*U*_1_	*U*_2_	*U*_3_	*U*_4_	*U*_5_	*U*_6_
*δ*_51_	0.241	0.234	0.230	0.251	0.229	0.229
*δ*_52_	0.241	0.225	0.230	0.251	0.229	0.229
*δ*_53_	0.241	0.234	0.230	0.251	0.229	0.237
*δ*_54_	0.234	0.234	0.230	0.251	0.229	0.229

**Step 6.** Calculate the relative weight $\delta_{pkq}^{*}(e_{q})$ of *O*_*p*_ to *O*_*k*_, and the result is shown in Tables 14–18.

**Table 14:** The relative weight of *O*_1_ to others.

	*U*_1_	*U*_2_	*U*_3_	*U*_4_	*U*_5_	*U*_6_
*δ*_12_	0.952	0.918	0.896	1.000	0.968	0.933
*δ*_13_	0.931	0.933	0.876	1.000	0.946	0.945
*δ*_14_	0.931	0.933	0.876	1.000	0.946	0.945
*δ*_15_	0.952	0.918	0.896	1.000	0.968	0.967

**Table 15:** The relative weight of *O*_2_ to others.

	*U*_1_	*U*_2_	*U*_3_	*U*_4_	*U*_5_	*U*_6_
*δ*_21_	0.961	0.933	0.914	1.000	0.913	0.945
*δ*_23_	0.961	0.933	0.876	1.000	0.913	0.945
*δ*_24_	0.931	0.933	0.876	1.000	0.913	0.945
*δ*_25_	0.952	0.954	0.896	1.000	0.968	0.967

**Table 16:** The relative weight of *O*_3_ to others.

	*U*_1_	*U*_2_	*U*_3_	*U*_4_	*U*_5_	*U*_6_
*δ*_31_	0.983	0.918	0.936	1.000	0.934	0.933
*δ*_32_	0.952	0.918	0.936	1.000	0.968	0.933
*δ*_34_	0.952	0.954	0.896	1.000	0.968	0.933
*δ*_35_	0.952	0.918	0.896	1.000	0.968	0.933

**Table 17:** The relative weight of *O*_4_ to others.

	*U*_1_	*U*_2_	*U*_3_	*U*_4_	*U*_5_	*U*_6_
*δ*_41_	0.983	0.918	0.936	1.000	0.934	0.933
*δ*_42_	0.983	0.918	0.936	1.000	0.968	0.933
*δ*_43_	0.961	0.897	0.914	1.000	0.913	0.945
*δ*_45_	0.983	0.918	0.896	1.000	0.968	0.967

**Table 18:** The relative weight of *O*_5_ to others.

	*U*_1_	*U*_2_	*U*_3_	*U*_4_	*U*_5_	*U*_6_
*δ*_51_	0.961	0.933	0.914	1.000	0.913	0.912
*δ*_52_	0.961	0.897	0.914	1.000	0.913	0.912
*δ*_53_	0.961	0.933	0.914	1.000	0.913	0.945
*δ*_54_	0.931	0.933	0.914	1.000	0.913	0.912

**Step 7**. Calculate the relative dominance *δ*_*pkq*_(*e*_*q*_) of *O*_*p*_ to *O*_*k*_ for attribute *q* by Eq (20), and the result is shown in Tables 19–23 (*α* = 0.88, *β* = 0.88, *θ* = 2.25), which derive from Tversky and Kahneman [83].

**Table 19:** The relative dominance of *O*_1_ to others.

	*U*_1_	*U*_2_	*U*_3_	*U*_4_	*U*_5_	*U*_6_
*δ*_12_	-0.380	-0.822	-0.866	-0.402	0.022	-0.856
*δ*_13_	-0.275	0.006	-1.084	0.003	0.020	0.004
*δ*_14_	-0.727	0.007	-1.198	0.002	0.022	0.013
*δ*_15_	-0.724	-0.268	-1.417	-0.885	0.023	0.009

**Table 20:** The relative dominance of *O*_2_ to others.

	*U*_1_	*U*_2_	*U*_3_	*U*_4_	*U*_5_	*U*_6_
*δ*_21_	0.005	0.010	0.010	0.006	-1.804	0.010
*δ*_23_	0.007	0.007	-0.592	0.004	-1.533	0.008
*δ*_24_	-0.403	0.014	-0.793	0.007	-1.611	0.004
*δ*_25_	-0.496	0.012	-0.702	-0.604	0.016	0.008

**Table 21:** The relative dominance of *O*_3_ to others.

	*U*_1_	*U*_2_	*U*_3_	*U*_4_	*U*_5_	*U*_6_
*δ*_31_	0.003	-0.535	0.012	-0.226	-1.654	-0.368
*δ*_32_	-0.534	-0.596	0.007	-0.306	0.019	-0.655
*δ*_34_	-0.775	0.008	-0.541	-0.314	0.006	-0.908
*δ*_35_	-0.665	-0.606	-0.901	-0.771	0.012	-0.490

**Table 22:** The relative dominance of *O*_4_ to others.

	*U*_1_	*U*_2_	*U*_3_	*U*_4_	*U*_5_	*U*_6_
*δ*_41_	0.009	-0.614	0.014	-0.157	-1.825	-1.087
*δ*_42_	0.005	-1.151	0.009	-0.524	0.020	-0.338
*δ*_43_	0.010	-0.658	0.006	0.004	-0.490	0.011
*δ*_45_	0.009	-0.656	-0.755	-0.973	0.009	0.009

**Table 23:** The relative dominance of *O*_5_ to others.

	*U*_1_	*U*_2_	*U*_3_	*U*_4_	*U*_5_	*U*_6_
*δ*_51_	0.009	0.003	0.016	0.012	-1.871	-0.708
*δ*_52_	0.006	-0.998	0.008	0.008	-1.318	-0.620
*δ*_53_	0.008	0.007	0.010	0.011	-0.999	0.006
*δ*_54_	-0.748	0.008	0.009	0.013	-0.759	-0.739

**Step 8.** Calculate the overall dominance degree by Eq (21)

*τ*(*O*_1_) = −9.770, *τ*(*O*_2_) = −8.410, *τ*(*O*_3_) = −10.780, *τ*(*O*_4_) = −9.113, *τ*(*O*_5_) = −8.625

**Step 9.** Rank the overall dominance degree *τ*(*O*_*p*_): *τ*(*O*_2_)>*τ*(*O*_5_)>*τ*(*O*_4_)>*τ*(*O*_1_)>*τ*(*O*_3_)

So, the alternative *O*_2_ is the best one.

### 4.2 Comparative analysis

In this section, we will take the advantage of classical TODIM method to compare with the improved CPT-TODIM under PHFSs. To make a better comparison, we use the same data from the Tables 1 to 3 and the attributes weight vector obtained from Step 4 is as follows:

$$e_{q}=(0.171,0.16,0.154,0.185,0.165,0.165)$$

The specific steps and results of the classical TODIM are shown as follows.

**Step 1.** We can calculate the weighting vector of attributes *e*_*q*_ and normalized group score matrix shown in Table 7 using the same method.

**Step 2.** Determine the dominance degree using Eq (23), and the result is shown in Tables 24–28.

**Table 24:** The dominance of *O*_1_ to others.

	*U*_1_	*U*_2_	*U*_3_	*U*_4_	*U*_5_	*U*_6_
*δ*_12_	-0.720	-1.127	-1.169	-0.734	0.127	-1.148
*δ*_13_	-0.594	0.063	-1.316	0.043	0.122	0.052
*δ*_14_	-1.031	0.068	-1.392	0.035	0.129	0.096
*δ*_15_	-1.035	-0.594	-1.541	-1.145	0.130	0.075

**Table 25:** The dominance of *O*_2_ to others.

	*U*_1_	*U*_2_	*U*_3_	*U*_4_	*U*_5_	*U*_6_
*δ*_21_	0.055	0.080	0.080	0.060	-1.731	0.084
*δ*_23_	0.066	0.067	-0.934	0.051	-1.585	0.072
*δ*_24_	-0.740	0.097	-1.105	0.070	-1.634	0.049
*δ*_25_	-0.832	0.089	-1.030	-0.918	0.107	0.070

**Table 26:** The dominance of *O*_3_ to others.

	*U*_1_	*U*_2_	*U*_3_	*U*_4_	*U*_5_	*U*_6_
*δ*_31_	0.045	-0.880	0.090	-0.527	-1.663	-0.709
*δ*_32_	-0.870	-0.936	0.064	-0.625	0.116	-0.983
*δ*_34_	-1.076	0.070	-0.892	-0.635	0.061	-1.183
*δ*_35_	-0.990	-0.948	-1.196	-1.062	0.091	-0.837

**Table 27:** The dominance of *O*_4_ to others.

	*U*_1_	*U*_2_	*U*_3_	*U*_4_	*U*_5_	*U*_6_
*δ*_41_	0.078	-0.952	0.095	-0.428	-1.759	-1.311
*δ*_42_	0.056	-1.355	0.076	-0.846	0.120	-0.672
*δ*_43_	0.082	-0.984	0.061	0.052	-0.829	0.087
*δ*_45_	0.080	-0.986	-1.075	-1.204	0.078	0.077

**Table 28:** The dominance of *O*_5_ to others.

	*U*_1_	*U*_2_	*U*_3_	*U*_4_	*U*_5_	*U*_6_
*δ*_51_	0.078	0.042	0.105	0.094	-1.773	-1.021
*δ*_52_	0.063	-1.251	0.070	0.076	-1.458	-0.950
*δ*_53_	0.075	0.068	0.082	0.087	-1.237	0.061
*δ*_54_	-1.051	0.070	0.074	0.099	-1.066	-1.049


$$\zeta_{q}(O_{p,}O_{k})=\{\begin{array}{cc} -\theta \sqrt{\frac{(\sum_{q=1}^{d}\left(e_{q}).d(\gamma_{pq},\gamma_{kq}\right)}{w_{j}}} & \mathrm{if}\;\gamma_{pq}-\gamma_{kq}<0\\ 0 & \mathrm{if}\;\gamma_{pq}-\gamma_{kq}=0\\ \sqrt{\frac{e_{q}.d(\gamma_{pq},\gamma_{kq})}{\sum_{q=1}^{d}e_{q}}} & \mathrm{if}\;\gamma_{pq}-\gamma_{kq}>0 \end{array}$$ (23)

**Step 3.** Obtain the overall dominance degree by Eq (21).

*τ*(*O*_1_) = −12.605, *τ*(*O*_2_) = −9.411, *τ*(*O*_3_) = −15.473, *τ*(*O*_4_) = −11.458, *τ*(*O*_5_) = −9.712

**Step 4**. Rank the overall dominance degree *τ*(*O*_*p*_): *τ*(*O*_2_)>*τ*(*O*_5_)>*τ*(*O*_4_)>*τ*(*O*_1_)>*τ*(*O*_3_).

So, the *O*_2_ is the best one.

At the same time, the improved CPT-TODIM under PHFSs is compared with PHFWA and PHFWG operators [15], Correlation Coefficients method [84], PHF-ORESTE method [85], PHF-TOPSIS method [86], PHF-COPRAS method [87] and PHF-MABAC method [88]. The comparative results are shown in Table 29.

**Table 29:** Order of different methods.

	Order
PHFWA operator [15]	*O*_2_>*O*_5_>*O*_4_>*O*_1_>*O*_3_
PHFWG operator [15]	*O*_2_>*O*_5_>*O*_1_>*O*_4_>*O*_3_
Correlation Coefficients method [84]	*O*_2_>*O*_5_>*O*_1_>*O*_4_>*O*_3_
PHF-ORESTE method [85]	*O*_2_>*O*_5_>*O*_4_>*O*_1_>*O*_3_
PHF-TOPSIS method [86]	*O*_2_>*O*_5_>*O*_4_>*O*_1_>*O*_3_
PHF-COPRAS method [87]	*O*_2_>*O*_5_>*O*_4_>*O*_1_>*O*_3_
PHF-COPRAS method [87]	*O*_2_>*O*_5_>*O*_4_>*O*_1_>*O*_3_

Comparing the results with existed eight decision methods, the obtained results are slightly different and the chosen best alternative is same. These nine given models have their given advantages. the improved CPT-TODIM under PHFSs is based on the value function of prospect theory, establishes the relative advantage function of one scheme compared with other schemes according to the psychological behavior of the decision-maker, and selects the best scheme according to the size of the advantage degree, so as to determine the best scheme. At present, the improved CPT-TODIM under PHFSs has been continuously improved and widely used in decision-making in various fields. However, the improved CPT-TODIM under PHFSs is compared with PT-TODIM under PHFSs [89], the same ranking order could be obtained. But, the main shortcoming of PT-TODIM under PHFSs [89] is: the amount of calculation is very large; the data needs to be decomposed into equal probability data, which further increases the calculation amount.

## 5. Conclusions

Digital inclusive finance directly promotes regional economic development by enhancing digital business capabilities within the banking industry, improving the business capabilities related to digital inclusive finance and expanding the scope of financial services. First, digital inclusive finance enhances the banking industry’s ability to provide inclusive financial services and reduces transaction costs. Due to the barriers to entry caused by government control, regional restrictions and capital accumulation, the development of China’s banking industry has been in a highly monopolistic state. A highly monopolistic market structure can cause low levels of efficiency and increased credit risks within banks, which directly affect the production and development of enterprises. The main carrier of digital inclusive finance implementation is banks, and the development of the banking industry to a certain extent restricts the development of digital inclusive finance. The rising degree of competition in the banking industry promotes the deepening of financial services and improves the digital inclusive finance capability of banks, which is conducive to improving the quality and diversity of banks’ services, providing more convenient and diverse inclusive financial products more directly to small and medium-sized enterprises, and reducing the disadvantaged groups’ "Financial exclusion" phenomenon. The theory of "financial exclusion" was first applied in the 1970s, meaning "a state in which certain groups in the financial system lack access to financial services for certain reasons, including some disadvantaged groups in society who lack adequate access to financial institutions, as well as access to financial products or services. This includes disadvantaged groups in society who lack adequate access to financial institutions and have difficulties and barriers in accessing financial products or services. In the development of the banking industry, the improvement of digital financial inclusion has, to a certain extent, reduced the phenomenon of "financial exclusion" and alleviated the problem of financing constraints of SMEs. Second, the development of digital inclusive finance improves the efficiency of information matching and reduces moral hazard and adverse selection in the process of investment and financing. The promotion and development of digital inclusive finance crosses the limits of traditional financial services, eliminates geographical barriers and time constraints, maximizes information sharing and service promotion, realizes the efficiency of information matching and information authenticity, thus reducing risks and enabling more long-tail customers to enjoy financial services, thus increasing the proportion of residents’ access to financial services, achieving better circulation of funds and promoting regional economic development. The development level of digital inclusive finance is a classical MAGDM. The classical TODIM neglect to distinguish the negative and positive attributes but focus on MADM in real number. Besides, it regards the initial weight vector of the attributes as the ultima weight vector. In this essay, we use the extended CPT-TODIM under PHFSs environment to solve MAGDM problem. First of all, the basic knowledge of the PHFE and extended TODIM are introduced. Moreover, the concept of entropy is used to calculate the weight of the attributes. In the end, the improved CPT-TODIM method is built for MAGDM under PHFSs environment. Finally, a numerical case for evaluating the development level of digital inclusive finance is given to testify the effectiveness of the new method with the comparation with the other methods’ results.

Based on the above findings, the following policy recommendations are proposed: First, enhance the digital inclusive finance capability of the banking industry. Large, medium and small banks focus on small and micro enterprises as well as long-tail customer groups, and establish special integrated services, risk management, assessment and evaluation mechanisms, etc. to enhance digital inclusive finance capabilities. Actively guide all kinds of institutions to use the Internet and other modern information technology to innovate products and service channels, reduce transaction costs, enhance service accessibility, and truly achieve "inclusive". Second, establish and improve the risk-sharing mechanism of digital inclusive finance, clarify the responsibilities and obligations of major banks, financial institutions and other individuals and institutions capable of providing digital inclusive financial services, and reduce the potential risks of individuals in the process of enjoying financial services. Third, increase the protection of financial consumers. Improve the system of protection of financial consumers’ rights and interests, widely carry out financial knowledge into ten thousand homes, campuses, communities and other publicity and popularization activities, use publicity films, public numbers and other channels to innovate publicity and education, establish a diversified mechanism for resolving financial consumer disputes, and govern violations of financial consumers’ rights and interests. Fourth, accelerate the construction of digital infrastructure, and fully promote and apply digital inclusive financial products and services. Accelerate the construction of infrastructure in the central and western regions, break through the digital barriers between regions, eliminate the barriers to the development of digital inclusive finance between regions, accelerate the narrowing of the digital divide between regions, and lay the foundation for inter-regional collaborative development. Fifth, continue to deepen the development of digital inclusive finance, expand the scope of its services, improve network coverage in small and medium-sized cities and villages, and further expand the digital inclusive finance user base, thereby promoting the coordinated economic development of all regions.
